The article "Multimedia System Design and Data Storage Optimization Based on Machine Learning Algorithm" was published in 2022. Journal: Comput Intell Neurosci.

# Multimedia System Design and Data Storage Optimization Based on Machine Learning Algorithm

**DOI:** 10.1155/2022/6426551

**Published:** 2022-08-01

**Authors:** Weiqiang Qi, Hongkai Wang, Tong Chen

**Affiliations:** State Grid Zhejiang Electric Power Corporation Information and Telecommunication Branch, Hangzhou, Zhejiang, China

## Abstract

With the advancement of science and technology, digital technology and Internet of Things network technology have been developed rapidly, and multimedia technology has also been widely used. Multimedia formats such as digital TV and elevator posters are shaking up traditional media. At the same time, many media operation models and multimedia technologies are combined to plan operational strategies, determine operational goals, and change the traditional media structure to achieve commercial profits and society benefit. However, due to limitations in the existing operating model or unreasonable technical solutions, it is not easy to maximize the value of multimedia technology. The XML-based database has been submitted, and it will carry out the business requirements of the transaction network and the business platform of the transaction network. Integrated management mechanism is analyzed and applied. The framework design includes parallel quota processing module, update processing module, result processing module, and storage library and database connection management module. The department runs multiple parts of the system together and completes the database. The development of cloud database is based on cloud computing. It can effectively fill the shortcomings and gaps of traditional database storage and processing, and it can also provide high-reciprocity databases to provide storage and management services. It has high reliability. Cloud servers use fair weighted rounding algorithms to achieve load balancing and use the in-memory database Redis to realize terminal data caching. After a comprehensive test of the system, the system can perform all functions normally, and it has good performance and stable operation.

## 1. Introduction

With the continuous development of the Internet of Things, the application of the Internet of Things is getting deeper and deeper, and the Internet of Things business is becoming more and more complex. Large-scale Internet of Things application systems and platforms that need to be supported by a transmission database continue to emerge [1]. However, due to the diversity and development of the Internet of Things services, many binary data principles have emerged in the Internet of Things due to the uniqueness of the process and the phasing of data source arrangements [2]. Internet services can meet some needs of some users. Although data has its own characteristics, it is difficult to access the data in the transmission database for business purposes, which leads to the phenomenon of “reading” information in business applications [3]. With the continuous development of services and applications, they inevitably create obstacles to work interaction and comprehensive solution analysis around data sources. Therefore, it is necessary to study and realize the operating mechanism of the Internet of Things and its database, and it has practical significance [4]. With the continuous development of cloud technology, cloud-related technologies can better provide users with corresponding services [5]. In today's information expansion, storing and processing a large amount of information pose a great challenge to traditional databases, so traditional data cannot well meet the processing needs of large amounts of information [6]. Therefore, when the cloud technology has developed to a certain level, the corresponding cloud database has begun to develop and obtain certain applications. Cloud database has a special function; it can provide users with more convenient information storage and processing functions, but if how to better serve users is mentioned, this requires the cloud database service management platform to handle it [7]. Therefore, the main purpose of this article is to demonstrate the core technology and implementation methods of the cloud database service management platform by simply summarizing the overall requirements and special design of the cloud database service management platform [8]. In the 21st century, with the development of multimedia technology, Internet technology, and digital technology, the multimedia technology called the fifth media has been rapidly developed and applied [9]. In fact, multimedia is not a new word. As early as 1967, the famous American researcher Goldmark put forward this concept, but at that time it was used to describe electronic video products, and it was a new form of media communication. Multimedia includes not only a series of traditional communication methods but also offline communication methods such as digital media [10]. The current media types are mainly Internet TV, architectural multimedia screens, digital TV, Internet newspapers, Weibo, and WeChat. Compared with traditional media, multimedia has the characteristics of more convenient information dissemination, more accurate information dissemination goals, higher dissemination rate, and richer dissemination content.

The article "Multimedia System Design and Data Storage Optimization Based on Machine Learning Algorithm" was published in 2022. Journal: Comput Intell Neurosci.

## 2. Related Work

With the widespread application of multimedia technology, people realize that the development of multimedia representation and operation platform fields is becoming more and more mature. In foreign countries, digital technology, IT technology, multimedia technology, and so forth started early, with a high level of information technology, and they were widely used in social life [11]. Literature introduces the main research background and significance of multimedia presentation system based on transaction network and cloud service technology and discusses relevant research status at home and abroad [12]. The literature combines the database heterogeneity of the USPIOT platform and the characteristics of the business data itself to conduct a comprehensive analysis of a problem and proposes an XML-based Internet database integration management mechanism, the crazy integration of the database and all functional components [13]. Literature creates an XML-based content database integrated management mechanism, uses JAVA, JDOM, and database connection technologies to perform integrated management of the content database, and then verifies its feasibility on usb [14]. Literature designed a unified management mechanism for IoT database based on XML by combining the heterogeneous characteristics of the USPIOT platform database and the characteristics of IoT business data itself. Literature discussed in detail the structural design and implementation of the cloud platform service system and at the same time introduced in detail the reverse proxy balance mechanism and the noncaching mechanism of the cloud platform service system [15]. Literature pointed out that, with the continuous development and universal application of multimedia technology, traditional media has received a huge impact. The effect of television in traditional media is significantly higher than that of newspapers, magazines, and radio. Literature pointed out that, with the widespread application of multimedia technology, the development of multimedia display and operation platform fields is becoming more and more mature, overseas digital technology, information technology, multimedia technology, and so forth started earlier, and the level of informatization is relatively high. The development of this field is relatively complete and has been widely used in social life.

## 3. Research on Internet of Things and Cloud Service Technology

### 3.1. Internet of Things Technology

The Internet of Things is not a fiction; it combines the research conclusions and results of researchers in many aspects. Kevin Ashton, who first proposed the concept of the Internet of Things, came up with the term Internet of Things during the research process of supply chain management, and the Internet of Things emerged following the research process of scholars on pervasive computing. The purpose of studying this computing technology is to allow people to incorporate more high-end technologies in their daily lives. Mark Weiser is the core of pervasive computing. It is described as follows: in the real world, there are many invisible monitors, sensors, execution calculators, and computing units. With the use of network connection, these devices can be integrated into the daily life environment. Thanks to the enhancement of technologies such as cloud computing and wireless sensor networks, the Internet of Things can provide customers with more flexible and reliable services. The Internet of Things has a large number of definitions. The RFID working group believes that the Internet of Things is a network based on standard communication protocols, with only one address and interconnected objects. European business departments are responsible for information activities, social processes, and business activities. They can interact with each other, and businesses can also interact with the external environment to obtain corresponding information and technology. Without any intervention, using autonomously stimulated behaviors to generate corresponding services can reflect real events and have a certain impact on them.

The article "Multimedia System Design and Data Storage Optimization Based on Machine Learning Algorithm" was published in 2022. Journal: Comput Intell Neurosci.

The Internet of Things system consists of three layers: network layer, detection layer, and application layer. Mainly related to the collection of various data, its components are mainly video capture equipment, various sensor equipment, wired sensors, and wireless sensor networks, including RFID. The sensing layer mainly has two technologies: one is short-distance transmission technology, and the other is controller and receiver technology. The access capability of the sensing layer will affect the realization of the Internet of Things. The network layer is built on the basis of the existing Internet and communication network. The core technologies of the network layer mainly include communication modules, existing communication technologies, and terminal technologies. Users can get corresponding services at the network layer as they wish, and, using the combination of wireless and wired and the cooperation between network technologies, users can choose the mode of intelligent connection to the network. The main function of the application layer is to realize the collection, sharing, intercommunication, cooperation, coordination, unification, analysis, and decision-making of the characteristics of items. The function is actually similar to the decision-making layer and the control layer of the Internet of Things. Because the ultimate goal of the Internet of Things is to serve people, and the application layer can complete the communication and interaction between people and objects, the function of the above two layers is mainly to collect the information of the items in a vague manner. Finally, the application layer realizes the overall compilation, summary, and arrangement of the data and then conducts consistent analysis and decision-making on the data. The purpose of the project is to realize different systems. Information is shared between different industries and different applications. Information is integrated to the greatest extent to provide customers with better services. Its related applications are mainly realized through the following aspects: intelligent logistics, intelligent transportation, and intelligent medical care. IoT architecture is shown in Figure 1.

The article "Multimedia System Design and Data Storage Optimization Based on Machine Learning Algorithm" was published in 2022. Journal: Comput Intell Neurosci.

The development of the Internet of Things and its related technologies determines the development areas and challenges of the Internet of Things. Nowadays, various regions have begun to have some small-scale related applications, but the Internet of Things is to realize the establishment of a plug-and-play intelligent body, which can complete the interaction with other intelligent objects in a specific operating environment. The core of this goal is to establish a consistent protocol and frequency band standard.

The bottleneck of the Internet of Things is the issue of technical standards. Because there may be differences in standards between countries, which affects the implementation process of the Internet of Things to a certain extent, the main goal at present is to find a standard that can be universally recognized. There are also problems with the protocol, because the Internet of Things is developed on the basis of the Internet, and its main foundation is the TCP/IP protocol. However, during the joining process, there are GPRS, wireless communication networks, text messages, sensors, and so forth. In the protocol, many connected things are encountered. Therefore, there must be a consistent basis for Internet access to things. In addition to the above problems, there are also some other problems: user safety issues. Because the Internet of Things realizes the communication between people and between people and things, information must be collected in this process, and information must be continuously exchanged between devices, so data security issues are getting more and more attention. The current bottleneck is how to protect users' personal privacy and security and address issues. If an IoT terminal wants to connect to the network, it must have an address. This realization process requires a large number of addresses, but the existing IPv4 is far from enough, and it takes a long time to transform from IPv4 to IPv6. As a network congestion problem, in the process of connecting sensor nodes to the network, it is inevitable to send and receive large amounts of data. But this time caused extreme network congestion, which in turn would have a predetermined impact on the quality of network service. Especially under the premise of a wireless environment, it is difficult to guarantee QoS. If there is still congestion in the network path, then this process will be even more difficult to achieve. The development route of the Internet of Things technology is shown in Figure 2.

The article "Multimedia System Design and Data Storage Optimization Based on Machine Learning Algorithm" was published in 2022. Journal: Comput Intell Neurosci.

### 3.2. Research on Cloud Service Technology

Cloud service is a service that integrates resources and services into the network so that users can use it through the Internet. Among them, “cloud” is a metaphorical term for the network and the Internet of Things. Therefore, cloud services are actually a type of service based on related services on the Internet of Things. When companies or individual developers actually develop and use cloud services, they can be used as cloud platforms provided by cloud service providers. Alibaba Cloud, Amazon Cloud AWS, Apple Cloud, Google's AppEngine service, and so forth are currently the world's most famous cloud service providers. The Aria Cloud used by this system is a cloud platform for all users. By renting, users can obtain cloud services at the lowest cost according to their needs. From the perspective of the development process of developers, program upgrades on the cloud platform are more convenient and faster than other conventional software upgrades. As a result, cloud services can be easily developed, and work efficiency can be reduced by reducing the workload. It can be seen that the development prospects of cloud service technologies are bright, and it is only a matter of time before they are widely promoted. As it deepens, at present, the application of cloud services is mainly realized from the three aspects of object association, security, and storage. In this project, the multimedia distribution system builds a server system based on cloud platform and a cloud link system with terminal devices.All working data and terminal data of the system are stored in the virtual disk of the cloud platform. In addition, with the support of the strong security provided by the cloud service provider, a series of protective measures have been taken within the system to ensure the absolute security of the system and data.

## 4. Related Research on Multimedia System and Database Design

### 4.1. Multimedia System Design Based on Internet of Things and Cloud Service Technology

The system needs to have the following functions:

1. Efficient, stable, and concise management and monitoring platform. The multimedia presentation system requires a management system for monitoring and managing terminals. The system must be able to log in and cannot access any content without an account and requires permission restrictions. The reason is that there are several brokers under the company and several stores, and each store is equipped with multimedia terminal equipment. Therefore, the system must be able to manage this information reasonably through relational design. Because of the relatively large fixed data such as terminals, the system must be able to import and export a large amount of efficient data. Terminals distributed across the country must be able to monitor the geographic location and operating status in real time through the management system. The results will be displayed on the map intuitively, and the advertiser's media file comment and preview function will be provided, and all video source files will be converted into one. The system must implement the specified transmission function to transmit random resources from media resources to random terminals nationwide. Media companies will collect fees from advertisers after video files are broadcast and paid regularly, and the system will regularly pay for all resources. The status of the terminal should be statistical information so that the company can understand the operating status of the entire system.
2. Safe, simple, and high-performance server platform. The media company does not provide the hardware equipment and storage space required to build a system server. Therefore, it is necessary to realize the safe and stable operation of the multimedia demonstration system by constructing a server system for the multimedia demonstration system based on the cloud platform.
3. Since a terminal playback platform with scalability and excellent user experience displays the playback terminal in front of the end user in the system, it is necessary to design a terminal playback system with a good user experience. It also provides weather forecast, temperature and humidity, PM_2.5_ measurement, and city location tracking functions, and when the wireless Internet connection is disconnected, Wi-Fi must be automatically reconnected. In addition, the broadcasting platform can also be upgraded to upgrade the remote control terminal broadcasting system.

The article "Multimedia System Design and Data Storage Optimization Based on Machine Learning Algorithm" was published in 2022. Journal: Comput Intell Neurosci.

The multimedia distribution system is a complete and complex Internet of Things system, including various issues, such as terminal management, media playback, server structure, terminal network, and data storage. Therefore, this task will be solved in the previous article. The development and implementation of the system is based on the demand analysis of the described project. The multimedia presentation system is divided into three parts. The development, design, and application arrangement of a single web project are divided into three parts, which are relatively separated in the form of development. But there is a close logical connection internally. Compared with a single person, web single management is divided into three parts: the system is the brain, the limb regeneration system is the limbs, and the cloud platform service system communicates with nerves and muscles at both ends to ensure safety and stability. In general, this system is a cloud connection system that combines the Internet of Things and cloud platforms. Partly, it has a complete triple structure of the Internet of Things. The overall structure of the system is shown in Figure 3.

1. Playback terminal: the playback terminal actually refers to the terminal of the Internet system of the object. Some information required by the device is actually its own playback data, and some information required by the playback terminal is environmental information, such as humidity, temperature, and NH3. In addition to implementing its own broadcasting function, the terminal must also transmit its own broadcasting data and environmental information (such as the collected temperature and humidity) to the server of the cloud platform through the device Wi-Fi or wired Internet.
2. Cloud platform server: the cloud platform server is the “link” of the entire system. It not only assumes the role of the system server but also serves as a platform for the operation of the web management system and a storage platform for all data. In addition, because it involves the entire system, the cloud platform in the system plays the role of cloud service, cloud storage, and cloud security, when the cloud platform accepts terminal playback requests. First, it is processed by the load balancing server and then sent to the web server. The web server responds to the request by calling the web application through the application program interface, so the cloud platform acts as the network and application layer.
3. Network management system: only the network management system receives the data information sent to the terminal and stores it in the database after being processed by the system user. The system user reproduces the terminal through the network management system and gives an opening instruction. Therefore, the web management system serves as the basis of the application, and the three parts of the system communicate with data through the network. Replaying the direct interviews with end users finally showed the users good usage results and informed the system usage. The cloud platform server is the entire system platform, which can ensure stable and efficient operation even under unexpected circumstances. The web management system is the part that directly interacts with users. Since it is responsible for the scientific management and integrated configuration of the multimedia presentation system, the broadcasting terminal and the cloud platform server are necessary factors of the system, and the web management system is the core of the entire multimedia.

The article "Multimedia System Design and Data Storage Optimization Based on Machine Learning Algorithm" was published in 2022. Journal: Comput Intell Neurosci.

As mentioned earlier, the multimedia distribution system implemented in this article is divided into three parts: web stage management system, cloud platform service system, and terminal broadcast system, which include optimization of performance and daily maintenance. This chapter introduces the design of the cloud platform service system in detail, but it is not limited to the main part of this chapter. The network management system and the terminal broadcasting system are relatively independent systems and are very important. In this project, the web-side management system is developed as a B/S framework, and the broadcasting software part of the terminal broadcasting system is developed as a C/S framework. There is no difference between the C/S and B/S structures. Its advantages and disadvantages are developing. Generally, large-scale system design must be considered in terms of server, data call, and mode conversion. Therefore, in a manner similar to this system, many large-scale systems in actual production are often developed by combining C/S and B/S, and the advantages and disadvantages of C/S and B/S structures are mainly discovered.

1. The C/S framework client in the functional area is realized through the system researcher's own design and can be used for subinterface control of the operating system. The actual system functions are file monitoring and direct communication. B/S browser supports a large number of frontal lobe structures, so it can display better data information, and, with the development of frontal lobe technology, Front Pro can implement some complex business theory functions.
2. In terms of applicability, the C/S structure requires users to install the client program and make corresponding arrangements at the same time. The C/S framework mainly implements functional changes by upgrading the existing client or reinstalling the user system. Based on the S frame web browser, all the functions of the system are realized. Therefore, when the system function changes, even if the system user does not perform an operation, the web application configured to the central server can be appropriately upgraded.
3. In the case of fusion, the fusion development of the C/S framework has its own uniqueness, and when the development is completed, the development of the fusion type is related to the operation, so the compatibility is very high. The B/S architecture relies on browsers to reflect all functions. Some major web browsers and some new web browsers have compatibility issues, so some new cutting-edge technologies may not be recognized as all web browsers.
4. The main process of B/S framework security is mainly processed by the server, and the browser mainly hides important data information, such as data display and user interaction. Some business logic and information data processing, transmission, and so forth are responsible for customers of the C/S structure. Therefore, a reasonable design size is required in data processing. The terminal playback system structure is shown in Figure 4.

The article "Multimedia System Design and Data Storage Optimization Based on Machine Learning Algorithm" was published in 2022. Journal: Comput Intell Neurosci.

### 4.2. Database Design Based on Internet of Things and Cloud Service Technology

With the increasing complexity of IoT applications and IoT services, relatively large IoT application systems or platforms that require structured database support continue to emerge. In this chapter, the unified management mechanism of the XML-based Internet of Things database is as follows: by combining the database heterogeneity of the USPIOT platform and the characteristics of the Internet of Things business data itself, an XML-based unified management mechanism of the Internet of Things database is designed. Mainly the following projects need to be completed:

1. Establish a global data model: for users of the Internet of Things platform, since the original data source data model with different structures is designed by different users based on different data models, there are bound to be some differences and collisions. To achieve collective nonprivate access to heterogeneous data sources without modifying the local mode, it is necessary to reconstruct a different data mode suitable for the whole world. Users can access the complete data mode, but, in order to obtain the actual data, they still need to obtain data from the default data source and need to establish a mapping between the global data mode and the local data mode.
2. Unified query model: with the rapid development of the Internet of Things, in order to meet the demand for more and more updates and more comprehensive data for the Internet of Things business, it is inevitable to access data in multiple databases. However, because the original data model and language of the basic database are different, this abnormally structured database system will maintain the original database system and ensure its own governance, and it is difficult to realize the exchange between multiple databases at the same time. Therefore, in order to support users to query the entire virtual database, a unified method can prevent different query access methods of existing structured data. Designing a search method is a relatively good way to achieve these interactions.
3. Maintain the independence of the heterogeneous structure database: under the premise that various existing tasks can work normally on the IoT platform, modify the existing DBMS as little as possible to protect the integrity and independence of each heterogeneous structure database.
4. Integration with the existing USPIOT platform: the USPIOT platform is an application scenario of the integrated management mechanism of the Internet of Things database based on XML. In order to integrate this mechanism with the existing USPIOT platform, it is necessary to establish a unified database management between the subordinate organization database and the database without changing the business functions of the existing USPIOT platform.

The article "Multimedia System Design and Data Storage Optimization Based on Machine Learning Algorithm" was published in 2022. Journal: Comput Intell Neurosci.

In the unified management of the database, the autonomy and heterogeneity of the underlying structure data will inevitably lead to conflicts with the data. Therefore, before the unified management of the database, the following structure data will conflict with each other. One of the first problems to be solved is the problem of data conflicts. In naming conflicts, there are two situations: conflicts with different names and conflicts with the same name. If two entities are the same or all or some of the attributes are the same, but the naming is different, our situation is called the same name conflict. Entity synonymous name conflict matching diagram is shown in Figure 5.

For different DBMS, the data types are different. For example, Oracle displays numbers as numbers, but Microsoft SQL Server data types are classified as specific examples, such as INT and numbers. In the database of this article, the XML/TSD data type is used in the design to uniformly manage the intermediate data, and the data type of the database is mixed and matched as the Opera/TSD data type.  Table 1 shows mapping relationship between database data types and XML Schema/TSD data types.

Keyword search technology is becoming a popular research topic in the database field. Currently, there are many methods to calculate the relational sequence of the database. Object-level keyword retrieval can better integrate the information scattered in each component. In this section, a new sequence strategy is proposed for the result sequence problem in the core search system of the relational database. At the same time, the correlation with health attributes has also been improved. The match degree is used to measure the content information of the key attributes in the object, and the correlation degree is used to measure the distribution of the nonkey attributes in the object. On the basis of this strategy, this paper proposes a method to understand the ranking search and ranking of database targets based on the content and value of nonkey attributes. Finally, combining the matching degree of key attributes and the correlation degree of nonkey attributes, a scoring function is given.

The article "Multimedia System Design and Data Storage Optimization Based on Machine Learning Algorithm" was published in 2022. Journal: Comput Intell Neurosci.

The sorting algorithm proposed in this section includes two parts: correlation based on nonkey attributes and correlation based on content. Finally, the two related score functions are added to obtain the total score function. According to the sorting algorithm, each query result will get a comprehensive correlation score, and then the result will be returned to the user in descending order of the score. The so-called key attribute refers to the attribute that contains the keyword, and the nonkey attribute refers to the attribute that does not contain the keyword. In relational databases, relativity refers to the degree to which an object is related to the search term. The relevance algorithm based on nonkey attributes includes two aspects: (a) weight and (b) relevance.

The correlation between the nonkey attributes in the object and the keyword *k*_*i*_ is calculated, and the relevant calculation formula is

(1) $$\begin{array}{c} \text{Correlation}\left(k_{i},ti_{z}\right)=\sum_{Auk\in X-AK_{i}}F\left(ti_{z}\left[Auk\right],k_{i}\right)\cdot W_{Auk}. \end{array}$$

(A) Weights use information entropy to measure the weights of nonkey attribute values. The calculation formula of the information entropy on the nonkey attribute *W* is as follows:
  (2) $$\begin{array}{c} E\left(Aw\right)=-\sum_{v_{i}\in \left[W\right]}^{m}p\left(w_{i}\right)\log_{b}p\left(w_{i}\right). \end{array}$$
According to the nature of information entropy, we define *W*_*Aw*_ as the weight of nonkey attribute values:
  (3) $$\begin{array}{c} W_{Aw}=\frac{1}{1+E\left(Aw\right)}. \end{array}$$
(B) There are a total of *m* database relational tables in the nonkey attribute-based correlation database. There are *n* tuples in the *i*-th relational table *T*_*i*_ = {*t*_*i*1_, *t*_*i*2_, *t*_*i*3_,…, *t*_*in*_}, *h* attributes *A*_*tt*_ = {*A*_*i*1_, *A*_*i*2_, *A*_*i*3_,…, *A*_*ih*_}. The user enters the keyword sequence *K* = {*k*_1_, *k*_2_, *k*_3_,…, *k*_*n*_}. If you search for *K*_*i*_ as a key, you can get a set of vowels *U*_*i*_ that contain *K*_*i*_ in the target. *T*_*i*_ = *x* vowel *T*_*i*_ = {*t*_*i*1_, *t*_*i*2_, *t*_*i*3_,…, *t*_*ix*_}. If the statistical information of set *U*_*i*_ is all *u* different nonkey key attribute values *A* = {*a*_1_, *a*_2_, *a*_3_,…, *a*_*u*_}. Define the number of occurrences of each nonkey attribute value of keyword *k*_*i*_ in the full attribute set (*A* + *B*) *k*_*i*_ as *f*_*j*_. The larger *f*_*j*_ is, the more important the attribute is relative to keyword *k*_*i*_. *f*_*j*_ may be relatively large, and the formula of *tf*_*j*_ is as follows:
  (4) $$\begin{array}{c} tf_{j}=1+\ln\;f_{j}. \end{array}$$

With greater number of occurrences of the attribute value *j* of the nonkey attribute, as the relevance to the related search word increases, we indicate the number of noncore attributes related to the relevant search word and the relevance as the relevance. We use *F*(*a*_*j*_, *k*_*i*_) to represent its correlation function:

(5) $$\begin{array}{c} F\left(a_{j},k_{i}\right)=R_{j}=\frac{tf_{j}}{x}=\frac{\left(1+\ln\;f_{j}\right)}{x}. \end{array}$$

The specific formula is as follows:

(6) $$\begin{array}{c} \text{Correlation}\left(k_{i},ti_{z}\right)=\sum_{Auk\in X-AK_{i}}\frac{\left(1+\ln\;f_{j}\right)}{x}\frac{1}{1+E\left(Aw\right)}. \end{array}$$

It is based on the relevance of the content. The relevance to the search keyword is calculated by calculating the median attribute value of the key attributes of all objects. By comparing the matching degree between the attribute value in the key attribute and the keyword, the content-based relevance is obtained. Content-based relevance measurement includes three aspects: standardized tuple frequency *stf*, standardized word frequency *nk*_*i*_*f*, and standardized keyword length *nkl*, calculated as follows:

(7) $$\begin{array}{c} \text{weight}\left(n_{ki}\right)=\frac{stf*nk_{i}f}{nkl}. \end{array}$$

(A) Standardized tuple frequency *stf* is calculated as follows:
  (8) $$\begin{array}{c} stf=\ln\left(\frac{T}{tf+1}\right). \end{array}$$
(B) The standardized word frequency *nk*_*i*_*f* is also called the standardized word frequency, and its calculation formula is as follows:
  (9) $$\begin{array}{c} nk_{i}f=1+\ln\left(kf\right). \end{array}$$
(C) The calculation formula of standardized keyword length *nkl* is as follows:
  (10) $$\begin{array}{c} nkl=h*kl+\left(1+h\right)*F\left(kl,sl,nkl\right). \end{array}$$

In practice, it is found that when *F*(*kl*, *sl*, *nkl*) = 60%, the ideal sorting effect can be obtained. The specific formula is as follows:

(11) $$\begin{array}{c} \text{weigh}\left(n_{ki}\right)=\frac{\ln\left(T/tf+1\right)*\left[1+\ln\left(kf\right)\right]}{h*F\left(kl,nkl\right)+\left(1+h\right)*kl}. \end{array}$$

Through the analysis of the total lighting function, the calculation method is obtained by calculating the score of each target as the correlation when calculating the alignment score. It consists of two parts: one is the score correlation (*k*_*i*_, *t*_*iz*_) based on nonkey attribute values, and the other is the score weight (*nk*_*i*_) based on the content relevance.

The article "Multimedia System Design and Data Storage Optimization Based on Machine Learning Algorithm" was published in 2022. Journal: Comput Intell Neurosci.

Based on content relevance, the scoring formula and summation formula of each object in the object set on keyword *k*_*i*_ are as follows:

(12) $$\begin{array}{c} \text{Score}\left(k_{i}\right)=\text{weight}\left(nk_{i}\right),\\ \text{Score}\left(K\right)=\sum_{i=1}^{t}{\text{Score}}_{w}\left(K_{i}\right). \end{array}$$

Based on the relevance of nonkey attributes, the scoring formula and the summation formula of each object on keyword *k*_*i*_ are obtained in the object set:

(13) $$\begin{array}{c} \text{Score}\left(k_{i},t_{iz}\right)=\text{Corr}\left(k_{i},t_{iz}\right),\\ \text{Score}\left(K,t_{h}\right)=\sum_{i=1}^{t}\text{Score}\left(k_{i},t_{iz}\right). \end{array}$$

The overall summation formula of the object is

(14) $$\begin{array}{c} {\text{Score}}_{\text{object}}=\alpha {\text{Score}}_{w}\left(K\right)+\left(1-\alpha \right){\text{Score}}_{\text{com}}\left(K,t_{h}\right). \end{array}$$

The services provided by the cloud database service management platform mainly include the following aspects: First, database users have the basic service rights to use the database, which is the main content provided by the cloud database service management platform. Second, when signing a contract or agreement with a user to specify the lease service of the cloud database, the cloud database service management platform needs to provide interface services that match the content of the agreement, which can greatly facilitate the further needs of the user. Of course, the user must verify information about the platform. Third, when multiple users request a cloud database, certain services can be allocated to the user, and the user must make adjustments, so as to meet the needs of most users for cloud databases. Fourth, provide users with a visual interface and enable them to query, add and delete their own services, and at the same time start, restart, and shut down services.

There are many algorithms suitable for two classifiers in machine learning algorithms, such as support vector machine algorithm and random forest algorithm. The following describes the support vector machine algorithm and the random forest algorithm. SVM uses the strategy of maximizing the interval to find the partitioning hyperplane that divides the two class samples in the space. In order to achieve the search for the indivisible linear segmentation problem and divide it into hyperplanes, the samples must be projected into a high-dimensional space with a kernel function.

(15) $$\begin{array}{c} K\left(x,x^{\prime }\right)=x^{r}x^{\prime },\\ K\left(x,x^{\prime }\right)={\left(x^{r}x^{\prime }\right)}^{d},\\ K\left(x,x^{\prime }\right)=\exp\left(\frac{-{\left\|x^{r}x^{\prime }\right\|}^{2}}{2\sigma^{2}}\right),\\ K\left(x,x^{\prime }\right)=\tanh\left(\beta x^{T}x^{\prime }+\theta \right). \end{array}$$

Decision tree is a learning method for classification and customization. These calculation methods require almost no data and are easy to understand and explain. In decision trees, information gain or Gini coefficient is usually used as an index to measure the purity of a sample set.

(16) $$\begin{array}{c} \text{Ent}\left(D\right)=-\sum_{k=1}^{n}p_{k}\log_{2}p_{k}. \end{array}$$

For the sample with feature *a*, the other samples are divided into the next step, and the division information obtained afterwards is defined as

(17) $$\begin{array}{c} \text{Gain}\left(D,a\right)=\text{Ent}\left(D\right)-\sum_{v=1}^{V}\frac{\left|D^{v}\right|}{\left|D\right|}\text{Ent}\left(D^{v}\right). \end{array}$$

The greater the size of the information gain, the higher the purity obtained by dividing the sample with the attribute *a*, and the better the division effect; the defect tree is more likely to have common problems, but the decision tree trained by this problem can be solved by the aggregation learning method.

The article "Multimedia System Design and Data Storage Optimization Based on Machine Learning Algorithm" was published in 2022. Journal: Comput Intell Neurosci.

As shown in Figure 6, learning is performed by using a series of decision tree algorithm results listed separately, and then these known results are sorted, summarized, and classified to obtain a learning result that is better than that of the decision tree alone. The first step of overall forest learning is to extract a random sample, which can be extracted from the training sample, generate each sample, and determine the best classification by voting on all decision trees.

SQL phrases are used to analyze phrases and extract digitized functions. This article uses an open-source lexical analyzer sqlparse, which can analyze 25 kinds of tokens, for convenience. This article defines the digitized features of SQL statements completely obtained from the token list output by sqlparse lexical analysis, counts the number of different tokens in the token list, and fills in the corresponding positions in the digitized feature vector. As shown in Table 2, example sentence 1 contains 1 DML, 1 Identifier, 1 IdentifierList, 1 Keyword, and 1 Where sentence. So its digitized feature vector is [0,0,0,0,0,0,0,1,0,0,0,0,1,1,0,1,0,0,0,0,0, 0,0,1,0]. Similarly, the digital feature of the SQL statement in example 2 is [0,0,0,0,0,0,0,2,0,0,0,0,2,1, 0,2,0,0,0,0,0,0,1,1,1].

The article "Multimedia System Design and Data Storage Optimization Based on Machine Learning Algorithm" was published in 2022. Journal: Comput Intell Neurosci.

To judge the performance of the classifier, comparison methods and performance indicators quoted from medical tests are often used. The method is to calculate the confusion matrix (CM) according to the classification results and the real labels, as shown in Table 3. The confusion matrix consists of four parts: the real number TP, the false negative number FN, the false positive number FP, and the true negative number TN. The real mother number is the sum of TP and FN. The number of true samples and negative samples is the sum of FP and TN; PO is the sum of TP and FP; the negative observation value NO is the sum of FN and TN, and the total number of factors is TE, FN, FP, and TN.

Performance indicators include true positive rate, false positive rate, accuracy, precision rate, recall rate, F1 index, false positive rate and missed positive rate, and the area under the ROC curve. The meaning of each performance index is introduced as follows:

(1) True positive rate (TPR): It is the ratio of the number of true positive samples to the number of positive samples, reflecting the accuracy of the classifier's detection of positive samples. The formula is
  (18) $$\begin{array}{c} \text{TPR}=\frac{\text{TP}}{\text{PE}}=\frac{\text{TP}}{\text{TP}+\text{FN}}. \end{array}$$
(2) False positive rate (FPR): it is the proportion of the number of false positive samples to the number of true negative samples. The higher the false positive rate, the higher the false positive rate of the classifier. The formula is as follows:
  (19) $$\begin{array}{c} \text{FPR}=\frac{\text{FP}}{\text{NE}}=\frac{\text{FP}}{\text{FP}+\text{TN}}. \end{array}$$
(3) Accuracy (*A*): it characterizes the overall detection accuracy of positive and negative events. The formula is
  (20) $$\begin{array}{c} A=\frac{\text{TP}+\text{TN}}{\text{TE}}=\frac{\text{TP}+\text{TN}}{\text{TP}+\text{FN}+\text{FP}+\text{TN}}. \end{array}$$

We use the training data set to obtain the two-SVM classifier and then test and analyze the data set in this classifier. The classifier outputs the probability in the range [0,1]. Select the default classification threshold (0.5 by default). When the score is greater than the threshold, it will be judged as 1, which means it is negative (normal SQL); when the score is less than the threshold, it will be judged as 0, which means it is positive (SQL injection). Finally, the classification results are compared with the real labels in the test training set, and the confusion matrix is obtained as shown in the third, fourth, fifth, and sixth columns of Table 4.

The article "Multimedia System Design and Data Storage Optimization Based on Machine Learning Algorithm" was published in 2022. Journal: Comput Intell Neurosci.

Calculate the performance indicators of the SVM classifier using four kernel functions, as shown in Table 5. When the classification decision threshold is set to the default value of 0.5, when the SVM uses linear kernel or radial kernel function, relatively high test accuracy can be obtained. However, in practical applications, the amount of SQL access to the database may be very large, leading to a large number of misjudgments. Too many misjudgments are obviously unsatisfactory. Next, search the classification decision threshold to explore the impact of the change of the decision threshold on the classification performance.

## 5. Conclusion

Nowadays, Internet technology and multimedia technology are rapidly spreading, and multimedia technology is gradually changing people's lifestyles. Therefore, this is not the era when people read newspapers and watch TV every day. In view of the shortcomings of single-version multimedia devices and Internet-based multimedia devices on the market, this paper constructs a multimedia presentation system that can be implemented at the current level. The project is realized by using the most mainstream language and software and hardware technology development under today's cloud platform and Internet of Things technology conditions, and the platform server system and the final playback system have been developed and designed. The Internet of Things is developing at an astonishing speed, which has led to a large number of various databases in various applications and services in the Internet of Things. The structure and storage of these data are different, which makes the Internet of Things business different. Data conversion, interaction, and unified processing have brought many problems and challenges. These heterogeneous databases are built into a unified global data model, which supports transparent access to the underlying heterogeneous database, but users do not need to view detailed information about the lower-layer heterogeneous structure database. Based on the actual problems in the existing USPIOT platform, this paper studies the unified data management mechanism of the Internet of Things, discusses in detail the related technologies of the unified data management middleware, and gives the specific design and implementation plan of the unified data management middleware. Based on the good design of the platform, users can monitor and manage terminal equipment distributed in various places in a short time, publish broadcast tasks, and perform real-time transmission. The cloud server system can receive a large number of requests, so that the system can run stably and safely. The system can be used stably and safely, and the terminal broadcasting system can display the surrounding environment and weather, while the equipment broadcasts the media, which can enhance the stability of the network.

The article "Multimedia System Design and Data Storage Optimization Based on Machine Learning Algorithm" was published in 2022. Journal: Comput Intell Neurosci.

## Figures and Tables

**Figure 1:** IoT architecture.

**Figure 2:** The development route of the Internet of Things technology.

**Figure 3:** Overall system architecture.

**Figure 4:** Terminal playback system.

**Figure 5:** Entity synonymous name conflict matching diagram.

**Figure 6:** Schematic diagram of the principle of the random forest algorithm.

**Table 1:** The mapping relationship between database data types and XML Schema/TSD data types.

Oracle data type	SQL Server data type	Sybase data type	XML Schema/ISDttiK type
UR	OUR	GUR	String
	MERIC	XIMERIC	Decimal

XDffiER	DECDLU	DECI1KL	Decimal
	SU^LLMOXEY	SAKLLMOXEY	—
	INT	IVT	Int
	SIULLIXT	SL4LLIXT	Short

FLOAT	FLQVT	FLOAT	—
	REAL	REAL	Float

DATE	DATETIME	WTETIME	Date
	SULLDATETIME	SU^LLDATCTIME	—
VAROUR2	VAROUR	XCHAR	String

XVAROUR2		XVAROUR	String
		VARCW	String
	BIT	BIT	Boolean

**Table 2:** Feature vector extraction example table.

Serial number	Feature	Meaning	Example l	Example 2
I	Assignment	Assignment word	0	0
2	Built-in	Built-in words	0	0
3	Case	Yu Kuang sentence marks old words	0	0
4	Comment	Annotation	0	0
5	Comparison	Comparison operator	0	0
6	CTE	Common agricultural sentences	0	0
7	DDL	Database definition	0	0
8	DML	Rescue database operation words	1	2
9	Error	Error	0	0
10	Float	Floating point	0	0
11	Function	Function	0	0
12	Hexadecimal	Hex save	0	0
13	Identifier	Identifier (field name)	0	2
14	IdentifierList	Identifier column clothing (uniform name column clothing)	0	0
15	Integer	Integer	0	0
16	Keyword	Guan Lv Ci	1	2
17	Operation	Operation scattered	0	0
18	Operator	Operator	0	0
19	Order	Order	0	0
20	Parenthesis	HI brackets	0	0
21	Placeholder	Placeholder	0	0
22	Punctuation	Punctuation	0	0
23	Single	Single line comment	0	1
24	Where	About fit word where	1	1
25	Wildcard	Wildcard (・)	0	I

**Table 3:** Definition of confusion matrix.

The true situation	Positive (p)	Clarity (N)	Sample meter
Positive (P)	True positive number (TP)	False brightness number (FN)	Number of positive samples (PE)
Negative (n)	Number of false positives (FP)	Truthfulness number (TK)	Number of brightness samples (NE)
Measurement statistics	Positive outlook (PO)	Negative observation (NO)	Total sample (TE)

**Table 4:** Confusion matrix of two-SVM classifier using different kernel functions.

	Formula	Linear kernel function	Transaction kernel function	Basic kernel function	Sigmoid function
True positive (TP)	—	219	227	219	210
False negative (FN)	—	13	5	13	*22*
False positive (FP)		8	39	6	*32*
True negative (TN)		188	157	190	164
Positive sample (PE)	TP + FN	232	232	232	232
Brightness sample (NE)	FP + TN	196	1%	1%	1%
Number of positive observations (POs)	TP + FP	227	266	225	242
Number of negative observations (NOs)	FN + TN	201	162	203	186
Total number of samples (TE)	PE + NE	428	428	428	428

The article "Multimedia System Design and Data Storage Optimization Based on Machine Learning Algorithm" was published in 2022. Journal: Comput Intell Neurosci.

**Table 5:** Different performance of two-SVM classifier using subcategory kernel function.

Kernel function	Viscosity	Accuracy rate	Gold check rate	F degree letter	Misjudgment rate	Missing rate	AUC
Linear kernel function	0.9509	0.9648	0.9440	0.9542	0052	0.0560	0.9727
Business item form	0.8972	0.6534	0.9784	0.9116	0.1466	0.0216	0.9804
Radial basis kernel function	0.9556	0.9733	0.9440	0.9584	0.0267	0.0560	0.9859
Sigmoid kernel function	03738	0.8678	0.9082	0.0886	0.1322	0.0948	0.8991

## Data Availability

The data used to support the ﬁndings of this study are available from the corresponding author upon request.
